The article "MicroRNA-424-5p Alleviates Isoflurane Anesthesia-Induced Neurotoxicity in Human Embryonic Stem Cell-Derived Neurons by Targeting FASN" was retracted in 2023. Reasons: unreliable results or conclusions; concerns about the data; concerns about the peer review; concerns about the citations.

# MicroRNA-424-5p Alleviates Isoflurane Anesthesia-Induced Neurotoxicity in Human Embryonic Stem Cell-Derived Neurons by Targeting FASN

**DOI:** 10.1155/2022/2517463

**Published:** 2022-07-13

**Authors:** Xiaojiao Gu, Wei Yue, Mingyu Xiu, Quanyun Zhang, Rufeng Xie

**Affiliations:** ^1^Department of Anesthesiology, The First People's Hospital of Lianyungang, Lianyungang 222000, China; ^2^Department of Anesthesiology, Women's Hospital of Nanjing Medical University, Nanjing Maternity and Child Health Care Hospital, No. 123, Tianfeixiang, Mochou Road, Nanjing 210004, China; ^3^Department of Pain Medical Center, Lianyungang Second People's Hospital, Lianyungang, 222000 Jiangsu, China

## Abstract

Isoflurane (ISO) is a type of anesthetic that might cause neurotoxicity in children. Although miR-424-5p is considerably downregulated in ISO-treated rat brain samples, its physiological role in ISO-induced neuronal injury in human embryonic stem cell-derived neurons remains unknown (hESC-derived neurons). miR-424-5p expression and fatty acid synthase (FASN) in ISO-treated hESC-derived neurons were tested via qRT-PCR. The amount of protein for Bax, Cleaved-caspase-8, Bcl-2, and FASN was investigated through western blot analysis. The viability and apoptosis of hESC-derived neurons were estimated through cell counting kit-8 assessment and TUNEL assay, accordingly. Superoxide dismutase, glutathione, and malondialdehyde levels were discovered via corresponding kits. The contents of inflammatory factors including interleukin-6 and tumor necrosis factor-*α* were examined by enzyme-linked immunosorbent assays. The combination between FASN and miR-424-5p was resolute via dual-luciferase reporter assessment. After exposure to ISO, induced neurotoxicity and a decreased miR-424-5p production were identified in hESC-derived neurons. Upregulation of miR-424-5p repressed ISO-induced apoptosis and mitigated ISO-induced inflammatory response and oxidative stress in vitro. FASN expression levels were reduced by elevation of miR-424-5p and upregulated after ISO treatment. Mechanically, FASN was directly targeted by miR-424-5p in hESC-derived neurons. Of note, the miR-424-5p elevation-suppressed neuronal apoptosis, inflammatory response, and oxidative stress were countered by upregulation of FASN.

## 1. Introduction

Plenty of newborns and pregnant women require anesthesia for diagnostic or operative targets [1, 2]. Due to the frequent use of anesthesia-related medicines, the challenges induced by anesthesia increase year by year [3]. Notably, the negative effects of prolonged or excessive exposure to anesthetics on the central nervous system, especially on memory and learning in children and infants, have been broadly represented [4, 5]. Isoflurane (ISO), as one of the most used inhalation anesthetics, simply crosses the placental barrier and decreases the regeneration of neuronal stem cells and inhibits the proliferation, sustenance, and development of human neural progenitor cells at clinically relevant concentrations [6–8]. In recent years, ISO-induced neuronal damage in the developing brain has received more and more attentions [9]. Animal studies have shown that ISO treatment leads to neuronal apoptosis, thus resulting in long-term cognitive dysfunction of rats [10]. These investigations illuminate that ISO can demonstrate potential toxic influences on neuronal progression. Anesthesia-associated neuronal apoptosis is one of the important mechanisms in anesthesia-induced nerve injury [11]. However, the mechanisms responsible for ISO-induced neuronal apoptosis and neural toxicity have not been completely clarified.

MicroRNAs, as a variety of small noncoding RNA molecules with 18 to 25 nucleotides, reduce mRNAs stability through adhering to the compatible pattern on the 3′-untranslated region (3′-UTR) of related mRNAs [12]. miRNAs are reported to functionally modulate plenty of biological procedures, including neuron differentiation, proliferation, and neuronal inflammation in both animals and humans [13]. It has been proved that miRNAs are implicated in the regulation of neurodegenerative disorders like spinal cord injury [14], Parkinson's disease [15], Alzheimer's disease [16], and subarachnoid hemorrhage [17]. In addition, numerous miRNAs are reported to control anesthesia-induced cognitive impairment. Downregulation of miR-106a alleviates the cognition-related impairments of mice subjected to ISO treatment [18]. miR-124 is confirmed to protect against sevoflurane-induced cognitive dysfunction via targeting the Capn4/NF-*κ*B signaling [19]. Recently, miRNAs have presented potential influence on the regulation of neuronal injury induced by ISO. miR-142-5p depletion alleviates ISO-inhibited neuron viability and mitigated ISO-stimulated neuron apoptosis [20]. Upregulation of miR-133b attenuates ISO exposure-induced apoptosis of hippocampal neurons [21]. Oxidative stress and neuroinflammation are crucial pathological procedures in neurological diseases [22]. Recent documents have manifested that oxidative stress and inflammatory response exert essential functions in ISO-induced neurons or rat models [23, 24]. Researchers found that dysregulated levels of oxidative stress indicators comprising superoxide dismutase (SOD), catalase (CAT), glutathione (GSH), malondialdehyde (MDA), and lactate dehydrogenase (LDH) may give rise to high risks of neuronal apoptosis in rats with Alzheimer's disease [25]. Additionally, ISO exposure results in the elevation of interleukin-1*β* (IL-1*β*), tumor necrosis factor-*α* (TNF-*α*), and interleukin-6 (IL-6) levels in hippocampal tissues of rats [26]. According to a previous report, miR-424-5p was verified to implicate in the modulation of neuronal apoptosis in ischemic stroke [27]. Furthermore, miR-424-5p displayed substantially decreased expression in ISO-treated rat brain samples [28].

The miR-424-5p influence on ISO-induced neurotoxicity of human embryonic stem cell-derived neurons (hESC-derived neurons) was the focus of this present exploration. It was speculated that miR-424-5p may alleviate ISO-induced neuron damage by suppression of oxidative stress and inflammatory response, which may present valuable therapeutic targets for treating ISO-induced neurotoxicity.

In vitro investigations have only confirmed the protective impact of miR-424-5p in ISO-treated hESC-derived neurons; in vivo assays are needed to confirm whether miR-424-5p has protective activity in ISO-treated animals. Second, because biological mechanisms are complicated, certain putative signaling pathways related with miR-424-5p in ISO-treated hESC-derived neurons should be investigated further.

The arrangements of the paper are as follows: Section 2 discusses the methods and materials.  Section 3 analyzes the result, and Section 4 evaluates the results.  Section 5 concludes the article.

## 2. Methods and Materials

### 2.1. Neural Differentiation of Human Embryonic Stem Cells

The human embryonic stem cell (hESC) line, human WA01 (H1) cell, was donated by WiCell (WiCell Research Institute, USA). The procedure for propagating and differentiating hESCs into neurons was based on previously published publications [29, 30], with minor modifications. During the night hours, mouse embryonic fibroblasts (MEFs) treated with mitomycin-C (AbMole, Shanghai, China) were plated in a plate with 6 wells precoated with 0.1 percent gelatin (Huijia Biotechnology, China) as a feeder layer.

HESCs were seeded in the plates containing 6 wells, and the conditions for cell culture were 5% CO_2_ and 37°C. To culture hESCs, stem cell propagation medium containing Dulbecco's modified Eagle's medium (DMEM; D6429, Sigma-Aldrich, St. Louis, USA) supplied by 10% fetal bovine serum (FBS; Sigma-Aldrich) and 1% penicillin streptomycin (Sigma Aldrich) was utilized. Cell passage was conducted upon the confluence which was up to 75% to 95%. The generation of neural progenitor cells (NPCs) was achieved through treating hESCs with neural progenitor milieu having DMEM/F12 (Sigma Aldrich) added with 20% knockout serum (Sigma Aldrich), 1% penicillin-streptomycin (Sigma Aldrich), 1 mM L-glutamine (Sigma Aldrich), 0.1 mM *β*-mercaptoethanol (Sigma Aldrich), and 1% nonessential amino acids (Sigma Aldrich) for 7 days. Subsequently, 5 ng/ml human recombinant basic fibroblast growth factor (bFGF, Sigma Aldrich) and the neuronal induction milieu including neural progenitor medium plus 1 mg/ml heparin (Sigma Aldrich) although without L-glutamine were employed to treat NPCs for 14 days. HESC-derived neurons were generated by collecting the rosettes from NPC cultivation and replated the rosettes in gelatin-coated plates containing 6 wells in a neuronal induction milieu with N2/B27 neural supplements (Sigma Aldrich) for ten to eighteen days.

### 2.2. ISO-Induced Neurotoxicity in hESC-Derived Neurons

ISO (Merck Millipore, USA) was used to concept ISO-induced cell model in vitro in this study. As illustrated in previous studies, hESC-derived neurons were processed with numerous quantities of ISO (0, 0.25%, 0.50%, 0.75%, 1.00%, 1.25%, and 1.50%) plus O_2_ (21%) and CO_2_ (5%) for 12 hours or similar quantity of ISO (1.00%) with O_2_ (21%) and CO_2_ (5%) for 0, 6, 12, 24, and 48 h [31, 32]. Briefly, hESC-derived neurons in 1.5 ml of cell culture medium with a density of 1 × 10^6^ were incubated in a plate containing 6 wells at 37°C. An anesthesia machine was used to deliver different concentrations of ISO with O_2_ (21%) and CO_2_ (5%) enclosed in a locked plastic container, in the incubator. The delivered concentrations of ISO, O_2_, and CO_2_ were continuously monitored by a Datex infrared gas analyzer (Puritan-Bennett, Tewksbury, USA).

### 2.3. Cell Transfection

miR-424-5p mimics were used for miR-424-5p overexpression while pcDNA3.1/FASN was used to elevate FASN expression. Genepharm (Shanghai, China) provided the miR-424-5p mimics, pcDNA3.1/FASN, and the related respective negative control (NC) mimics and empty pcDNA3.1. The abovementioned oligonucleotides were transfected into hESC-derived neurons treated with or without ISO using Lipofectamine 2000 (Invitrogen, USA). Neurons transfected with random sequences of oligonucleotides by Lipofectamine 2000 served as the negative controls. Twenty-four hours later, the transfected samples were collected for the follow-up experiments.

### 2.4. Quantitative Real-Time Polymerase Chain Reaction (qRT-PCR)

The qRT-PCR was executed as the method demonstrated in the last report [33]. Total RNA of hESC-derived neurons was extracted through TRIzol reagent (Invitrogen, USA) as instructed by the product manuals. The reverse transcription kit (QIAGEN, Germany) was applied for the reverse transcription of total RNA into complementary DNA (cDNA). The qRT-PCR was working to assess the quantities of miRNAs or mRNAs via the SYBR Green Master Mix (Vazyme Biotech Co., Ltd, China). The thermal cycling conditions for qRT-PCR was 95°C × 5 min, 40 cycles of 95°C × 30 s, 60°C × 30 s, and 72°C × 1 min. The PCR primers are shown as follows: miR-424-5p forward: 5′-GCCAGCAGCAATTCATGT-3′, reverse: 5′-TATGGTTTTGACGACTGTGTGAT-3′; FASN forward: 5′-CAACCTCTCCCAGGTATGC-3′, reverse: 5′-TGCTGATGATGGACTCCAG-3′; glyceraldehyde-3-phosphate dehydrogenase (GAPDH) forward, 5′-TGCACCACCAACTGCTTAGC-3′, reverse: 5′-GGCATGGACTGTGGTCATGAG-3′; U6 forward: 5′-CCCCTGGATCTTATCAGGCTC-′, reverse: 5′-GCCATCTCCCCGGACAAAG-3′. GAPDH served as internal reference for mRNA while U6 functioned as internal reference for miRNA. The StepOnePlus™ software (Thermo Fisher Scientific, USA) was employed for analyzing the miRNA or mRNA expression which were then evaluated by the 2^−*ΔΔ*Ct^ approach [34].

### 2.5. Western Blot Analysis

RIPA buffer (V900854, Merck & Co Inc, USA) was employed for extracting the entire protein samples from hESC-derived neurons for half an hour. The collected lysates centrifuged at 12,000 × g for 15 minutes yielded 35 micrograms of protein which was divided through 10% sodium dodecyl sulfate-polyacrylamide gel electrophoresis (SDS-PAGE; KL81205-30, KLANG, Shanghai, China), followed by being moved to 0.22 *μ*m polyvinylidene difluoride (PVDF) membranes (3010040001, Merck & Co Inc) for 2 h. After being blocked with 5% nonfat milk in Tris-buffered saline plus 0.02% Tween-20 (TBST) at 37°C for 1.5 hours, incubation of membranes was done with the primary antibodies versus Bax (1/1000, #5023, CST), Cleaved-caspase-8 (1/1000, #9496, CST), Bcl-2 (1/1000, #15071, CST), FASN (1/1000, #3180, CST), and GAPDH (1/1000, #2118, CST) during the night hours in a 4°C refrigerator. After that, membranes were treated for one hour at 37°C by horseradish peroxidase-conjugated (HRP) secondary antibodies. The enhanced chemiluminescence (ECL) system (RPN2108, Cytiva, Shanghai, China) was used for the observation of all protein bands that were normalized to GAPDH and quantified by ImageJ software (NIH, Bethesda, USA) [35].

### 2.6. Cell Counting Kit-8 (CCK-8) Assay

The hESC-derived neuron survival was examined through CCK-8 assessment as instructed by the manufacturer. After inoculating hESC-derived neurons (5 × 10^3^ cells/well) into the plates containing 96 wells, the transfected cells were processed with or without ISO and then cultured by 10 *μ*l of CCK-8 solution (CK04, SciencBio, Beijing, China) at 37°C for another 4 h. Microplate reader (Bio-Rad, USA) was adopted for determining the optical density (OD) at 450 nm.

### 2.7. Terminal Deoxynucleotidyl Transferase dUTP Nick End Labeling (TUNEL) Staining

As per the instructions of the in situ cell death detection kit (Roche, Basel, Switzerland), DNA fragmentation was detected and TUNEL staining assessment was performed. In brief, hESC-derived neurons with a density of 1 × 10^5^ cells in each well were placed in a plate containing 6 wells. 24 hours later, the cultivated neurons were washed with cold PBS, fixed by 4% paraformaldehyde, and were permeated with 0.25% Triton X-100, respectively. Then, TUNEL reaction buffer was adopted to process the neuron samples for 01 hour and 4′,6-diamidino-2-phenylindole (DAPI) solution (Invitrogen) was utilized to counterstain all nuclei. Observation of the positive apoptotic neurons was achieved by using a microscope.

### 2.8. Enzyme-Linked Immunosorbent Assay (ELISA)

According to instructions of IL-6 kit (Y-S Biotechnology, Shanghai, China) and TNF-*α* kit (Has Biotech, Shenzhen, China), the contents of TNF-*α* and IL-6 were estimated via ELISA. In brief, hESC-derived neurons were inserted with NC mimics, miR-424-5p mimics, or miR-424-5p mimics+FASN and were then treated with 1.00% of ISO for 12 h. After being washed by PBST (Sigma, USA), the collected supernatants were added into the plates containing 96 wells which were coated with primary antibodies and cultivated at 37°C for 2 h. Subsequently, HRP-conjugated secondary antibodies were put into plates and further cultured for 1 hour at 37°C. After adding 2 mol/l sulfuric acid solution to each well to stop the reaction, an ELISA reader (Sigma) was instantly used for the observation of the absorbance at 570 nm.

### 2.9. Measurement of Superoxide Dismutase (SOD) Activity and Decreased Glutathione (GSH) and Malondialdehyde (MDA) Quantity

Transfected hESC-derived neurons were accumulated and the SOD, GSH, and MDA quantities were examined with SOD assay kit (KTB1030-1, Abbkine, China), GSH assessment kit (KTB1600-2, Abbkine, China), and MDA assessment kit (KTB1050-2, Abbkine, China) as instructed by the manufacturer's protocols.

### 2.10. Dual-Luciferase Reporter Assay

The mutant (Mut) 3′-UTR and wild-type (WT) sequences of FASN were intensified and placed in luciferase reporter pmirGLO (Promega, US) to construct FASN-Wt and FASN-Mut vectors. Lipofectamine 2000 (Promega, US) was used for the cotransfection of FASN-Wt or FASN-Mut with miR-424-5p mimics or NC mimics in hESC-derived neurons. After 48 h, the luciferase activities of transfected hESC-derived neurons were examined by employing a luciferase detection kit (K801-200; BioVision Milpitas, USA).

### 2.11. Statistical Analysis

GraphPad Prism computer program, version 7.0 (San Diego, US), was applied to for carrying out the statistics. Biorepeats were run in triplicate, and the obtained experimental outcomes are demonstrated as mean ± standard deviation. For comparing the 02 groups, unpaired two-tailed Student's *t* test was employed. Discrepancies between various groups were scrutinized by 1-way ANOVA accompanied by Tukey's post hoc analysis. Significance was denoted as *p* value lower than 0.05.

## 3. Results

### 3.1. ISO Induces Neurotoxicity and Downregulation of miR-424-5p

miR-424-5p is validated for being decreased in ISO-treated rat brain samples. To ascertain miR-424-5p expression in ISO-treated hESC-derived neurons, qRT-PCR was conducted, and the results illustrated that after treating hESC-derived neurons by different doses of ISO (0, 0.25%, 0.50%, 0.75%, 1.00%, 1.25%, and 1.50%) for 12 h, miR-424-5p expression displayed a significant downward trend (Figure 1(a)). Subsequently, miR-424-5p expression was tested in hESC-derived neurons treated with 1.00% of ISO for 0, 6, 12, 24, and 48 h. Furthermore, miR-424-5p expression was time-dependently suppressed by 1.00% of ISO (Figure 1(b)). The effects of various ISO concentrations (0, 0.25 percent, 0.50 percent, 0.75 percent, 1.00 percent, 1.25 percent, and 1.50 percent) on the survival of hESC-derived neurons were then investigated. CCK-8 analysis revealed that ISO decreased the survival of hESC-derived neurons in a dose-dependent manner, demonstrating that ISO stimulation caused neurotoxicity in hESC-derived neurons (Figure 1(c)). Similarly, the survival of hESC-derived neurons was decreased as time passed after 1.00 percent ISO treatment, and in the subsequent studies, 1.00 percent ISO was used to grow the hESC-derived neurons for 24 hours (Figure 1(d)). Finally, ISO produced neurotoxicity in hESC-derived neurons, and ISO stimulation decreased miR-424-5p expression in a dose- and time-dependent manner.

### 3.2. miR-424-5p Overexpression Inhibits ISO-Induced Cell Apoptosis

To probe the physiological role of miR-424-5p in ISO-mediated apoptosis of hESC-derived neurons, miR-424-5p transfection with NC mimics was executed. As displayed in Figure 2(a), compared with hESC-derived neurons transfected with NC mimics, miR-424-5p production was significantly elevated following miR-424-5p mimic transfection. Importantly, ISO notably decreased miR-424-5p production in hESC-derived neurons, while this effect was altered by miR-424-5p mimics. Afterwards, viability of hESC-derived neurons was tested by performing CCK-8 assay. Results manifested that miR-424-5p-augmented production countered the suppressed viability of ISO-stimulated hESC-derived neurons (Figure 2(b)). In subsequent assays, the proteins (Bax, Cleaved-caspase-8, and Bcl-2) associated with cell apoptosis were appraised through western blot assessment. It was discovered that protein amount of Bax and Cleaved-caspase-8 enhanced by ISO were reduced by upregulated miR-424-5p. However, transfection of miR-424-5p mimics rescued the suppression of ISO treatment on Bcl-2 protein level (Figure 2(c)). TUNEL assay further illuminated that ISO stimulation-induced promotion on cell apoptosis was suppressed via overexpressed miR-424-5p (Figure 2(d)). Thus, it was concluded that ISO-induced cell apoptosis was inhibited through miR-424-5p elevation.

### 3.3. miR-424-5p Upregulation Alleviates ISO-Induced Inflammatory Response and Oxidative Stress

miR-424-5p has been illuminated for the inhibition of inflammatory response and regulate oxidative stress [36, 37]. Therefore, it was aimed at investigating whether miR-424-5p suppresses inflammatory reactions and modulates oxidative stress in ISO-induced hESC-derived neurons. ELISA was implemented for examining the quantities of inflammatory mediators (IL-1 and TNF-*α*). The experimental data illuminated that ISO treatment-mediated promotion on the TNF-*α* and IL-6 levels was partially abolished by miR-424-5p upregulation (Figure 3(a)). Subsequently, the influence of miR-424-5p mimics on oxidative stress in hESC-derived neurons was examined. It was observed that ISO treatment decreased the amount of GSH and SOD while it enhanced the MDA level. Nonetheless, these impacts were altered by upregulation of miR-424-5p (Figure 3(b)). Achieved observations demonstrate that overexpressed miR-424-5p ameliorated inflammatory response and oxidative stress induced by ISO in hESC-derived neurons.

### 3.4. miR-424-5p Targets FASN in hESC-Derived Neurons

Seven potential downstream targets (PAPPA, FASN, UNC80, FGF2, TNRC6B, PTPN4, and PHF19) that may have binding sequences with miR-424-5p were identified using bioinformatics analysis utilising the miRDB website with the screening condition of target score = 100. Only FASN mRNA expression was downregulated in hESC-derived neurons after the insertion of miR-424-5p mimics, according to qRT-PCR analysis, while the other mRNAs showed no significant change when miR-424-5p production was raised (Figure 4(a)). As a result, it was postulated that miR-424-5p could target FASN. The level of protein for FASN was investigated using a western blot to confirm this theory. As a result, FASN protein level was notably reduced in hESC-derived neurons after miR-424-5p mimics transfection (Figure 4(b)). Protein and mRNA of FASN which presented the increased levels were also observed in ISO-treated hESC-derived neurons (Figure 4(c)). According to StarBase, miR-424-5p was estimated to have a site of binding for FASN (Figure 4(d)). To prove the combination between FASN and miR-424-5p further, luciferase reporter assessment was applied. miR-424-5p mimics substantially decreased luciferase activity of FASN-Wt, although no notable change was observed in the FASN-Mut group (Figure 4(e)). Here, it was determined that FASN was directed targeted by miR-424-5p in hESC-derived neurons.

### 3.5. Elevation of miR-424-5p Attenuates Neuron Apoptosis, Inflammatory Response, and Oxidative Stress by Targeting FASN

Several restoration studies in ISO-stimulated hESC-derived neurons were carried out to investigate the impact of the miR-424-5p/FASN axis on neuronal apoptosis, inflammatory response, and oxidative stress. Transfecting pcDNA3.1/FASN into ISO-treated hESC-derived neurons increased FASN protein and mRNA expression (Figure 5(a)). The CCK-8 experiment revealed that increasing FASN inhibited miR-424-5p-overexpressing hESC-derived neurons from proliferating (Figure 5(b)). Furthermore, FASN overexpression reversed the inhibition of apoptosis in ISO-treated hESC-derived neurons caused by miR-424-5p mimics (Figure 5(c)). Overexpressed FASN also saved the inhibitive property of miR-424-5p elevation on IL-6 and TNF-*α* level (Figure 5(d)). Furthermore, as presented in Figure 5(e), elevation of FASN reversed the promotive impacts of miR-424-5p mimics on SOD and GSH quantities, while reversing the inhibitive effect of miR-424-5p upregulation on the MDA levels. Achieved findings ascertained that miR-424-5p elevation alleviated neuron apoptosis, inflammatory response, and oxidative stress in ISO-stimulated hESC-derived neurons by suppression of FASN.

## 4. Discussion

To date, a large portion of infants and children require anesthesia surgery during treatment procedures, which may affect neuronal function and development of brains [38]. In addition, approximately 30% of adults aged 65 or older receive some form of anesthesia each year in developed countries, but inhalation of anesthetics influences the neuropathogenesis of patients to a great extent [39, 40]. miRNAs have been validated to be involved in anesthesia-mediated neurotoxicity [41]. HESC-derived neurons are broadly employed for constructing anesthetic-induced models in vitro [42]. Therefore, the task and molecular strategy of miR-424-5p on anesthesia-induced neurotoxicity by constructing ISO-induced hESC-derived neurons in vitro were investigated.

A growing number of studies have shown that miRNAs are linked to anesthesia-induced neurotoxicity [43]. According to a recent study, miR-424-5p is implicated in ropivacaine-mediated cell growth, and silencing miR-424-5p counteracts ropivacaine-induced cell development and promotes cell death [44]. It is worth noting that miR-424-5p has been shown to have low expression in ISO-treated rat brain tissues [28]. This study consistently found downregulated expression of miR-424-5p in ISO-stimulated hESC-derived neurons. Moreover, it was also found that ISO treatment led to the repressed neuron viability and elevated neuron apoptosis presented by the higher number of TUNEL positive cells and enhanced Bax and Cleaved-caspase-8 protein levels and also the weakened Bcl-2 protein production, but miR-424-5p overexpression partially eliminated these effects. It was identified that oxidative stress and neuroinflammation are vital pathological procedures in neurological diseases [45]. The miR-424-5p effect on oxidative stress and inflammation response has been detected in lipopolysaccharide-induced acute lung injuries that miR-424-5p hinders LPS-driven injuries through decreasing the levels of LDH, ROS, MDA, TNF-*α*, IL-1*β*, and IL-1*β* [37]. Here, the miR-424-5p effect on oxidative stress and inflammation response in ISO-treated hESC-derived neurons is discovered. Results illustrated that elevation of miR-424-5p repressed the TNF-*α* and IL-6 in ISO-treated hESC-derived neurons. Similarly, overexpressed miR-424-5p altered the levels of oxidative stress markers shown as an enhancement in GSH and SOD levels and reduced levels of MDA in ISO-treated hESC-derived neurons. The findings illuminated that upregulation of miR-424-5p inhibited ISO-induced inflammation response and oxidative stress in hESC-derived neurons.

Although new evidence suggests that miR-424-5p plays a regulatory role in a variety of physiopathological processes, the exact biological mechanism by which it works in ISO-induced hESC-derived neurons is unknown. Understanding how miR-424-5p genes affect ISO-induced hESC-derived neurons requires determining which miR-424-5p genes should be targeted. In this study, through searching online website miRDB, fatty acid synthase (FASN), which presented downregulated production in hESC-derived neurons by the transfection of miR-424-5p mimics, was predicated to be the downstream target of miR-424-5p. FASN, as a central lipogenic enzyme that produces free fatty acids, was determined to interact momentarily with protrudin [46]. It has been reported that FASN is involved in the myelination and remyelination in the central nervous system [47]; however, almost nothing is understood regarding its molecular processes in anesthesia-induced neurotoxicity. In this investigation, by performing dual-luciferase reporter assay, FASN was validated to be directly targeted by miR-424-5p. In addition, it was found that the production of FASN at levels of mRNA and protein in hESC-derived neurons after ISO treatment was upregulated. Importantly, it was discovered that miR-424-5p overexpression-triggered repression on inflammation response and oxidative stress was partially abrogated by upregulation of FASN.

Briefly, the findings of the current analysis designated that miR-424-5p alleviates ISO anesthesia-driven neurological damage in hESC-derived neurons by suppression of apoptosis, inflammation response, and oxidative stress via downregulating FASN. As far as we know, this is the unprecedented research for probing into the purpose of miR-424-5p/axis in ISO-induced neurotoxicity in hESC-derived neurons, which may deliver implications for the treatment ISO-induced neurotoxicity. However, there are some limitations in this research. First, the protective effect of miR-424-5p in ISO-treated hESC-derived neurons was just validated in in vitro experiments, and in vivo assays are necessary to further verify if miR-424-5p exhibits the protective activity in ISO-treated animals. Second, due to the complexity of biological mechanisms, some potential signaling pathways associated with miR-424-5p in ISO-treated hESC-derived neurons deserve further exploration.

## 5. Conclusion

miR-424-5p alleviates ISO-induced neurotoxicity, inflammatory response, and oxidative stress in hESC-derived neurons by downregulating FASN.

## Figures and Tables

**Figure 1:** ISO induces neurotoxicity and downregulation of miR-424-5p. (a) miR-424-5p expression in hESC-derived neurons after treatment with increased ISO quantities for 12 hours was examined by qRT-PCR. (b) miR-424-5p expression in hESC-derived neurons was administered with 1.00% of ISO for various times (0, 6, 12, 24, and 48 h) by qRT-PCR. (c) After treatment of hESC-derived neurons with increased doses of ISO for 12 h, CCK-8 was performed to determine cell survival. (d) The viability of hESC-derived neurons was detected after treatment with 1.00% of ISO for 0, 6, 12, 24, and 48 h by CCK-8 assay. ^∗^*p* < 0.05, ^∗∗^*p* < 0.01, and ^∗∗∗^*p* < 0.001.

**Figure 2:** miR-424-5p overexpression inhibits ISO-induced cell apoptosis. HESC-derived neurons were treated with or without 1.00% of ISO for 24 h and divided into four groups: Con+NC mimics, Con+miR-424-5p, Isoflurane+NC mimics, and Isoflurane+miR-424-5p. (a) miR-424-5p overexpression in hESC-derived neurons. (b) The viability of hESC-derived neurons was detected via CCK-8 assay. (c) Apoptosis proteins (Bax, Bcl-2, and Cleaved-caspase-8) by western blot assessment. (d) The impacts of miR-424-5p elevation on ISO-mediated apoptosis of hESC-derived neurons was detected by TUNEL assessment.^∗^*p* < 0.05, ^∗∗^*p* < 0.01, and ^∗∗∗^*p* < 0.001.

**Figure 3:** miR-424-5p upregulation alleviates ISO-induced inflammatory response and oxidative stress. After treating the hESC-derived neurons with or without 1.00% of ISO for 24 h, the follow-up experiments were conducted. (a) ELISA was employed for the evaluation of IL-6 and TNF-*α* levels after transfection of NC mimics or miR-424-5p mimics. (b) The levels of SOD, GSH, and MDA in hESC-derived neurons after transfection were evaluated through the relative kits. ^∗^*p* < 0.05, ^∗∗^*p* < 0.01, and ^∗∗∗^*p* < 0.001.

**Figure 4:** miR-424-5p targets FASN in hESC-derived neurons. (a) The effect of miR-424-5p mimics on mRNA levels of PAPPA, FASN, UNC80, FGF2, TNRC6B, PTPN4, and PHF19 through qRT-PCR. (b) The protein quantity of FASN in transfected hESC-derived neurons by western blot. (c) Protein and mRNA quantity for FASN in hESC-derived neurons processed with or without 1.00% of ISO for 24 h was ascertained through qRT-PCR and western blot, accordingly. (d) The position of binding among miR-424-5p and FASN predicted from StarBase. (e) Luciferase activity of FASN-Wt or FASN-Mut in hESC-derived neurons inserted with NC mimics or miR-424-5p mimics was assessed through the luciferase reporter assessment. ^∗∗∗^*p* < 0.001.

**Figure 5:** Upregulation of miR-424-5p attenuates neuron apoptosis, inflammatory response, and oxidative stress by targeting FASN. After hESC-derived neurons were subjected to 1.00% of ISO for 24 h, the following rescue assays were performed. (a) Overexpression efficacy of FASN. (b) The viability of hESC-derived neurons was detected via CCK-8 assay in NC mimic, miR-424-5p mimic, and miR-424-5p+FASN groups. (c) TUNEL assay was implemented to appraise apoptosis in the abovementioned groups. (d) ELISA was used for the assessment of IL-6 and TNF-*α* levels after transfection of NC mimics, miR-424-5p mimics, or miR-424-5p+FASN. (e) Indicated plasmids were transfected into hESC-derived neurons to test the activities of SOD, GSH, and MDA. ^∗^*p* < 0.05, ^∗∗^*p* < 0.01, and ^∗∗∗^*p* < 0.001.

## Data Availability

Data will be provided upon request to the authors.
